The article "A Novel Hybrid Deep Learning Model for Metastatic Cancer Detection" was published in 2022. Journal: Comput Intell Neurosci.

# A Novel Hybrid Deep Learning Model for Metastatic Cancer Detection

**DOI:** 10.1155/2022/8141530

**Published:** 2022-06-24

**Authors:** Shahab Ahmad, Tahir Ullah, Ijaz Ahmad, Abdulkarem AL-Sharabi, Kalim Ullah, Rehan Ali Khan, Saim Rasheed, Inam Ullah, Md. Nasir Uddin, Md. Sadek Ali

**Affiliations:** ^1^School of Management Science and Engineering, Chongqing University of Post and Telecommunication, Chongqing 400065, China; ^2^Department of Electronics and Information Engineering, Xian Jiaotong University, Xian, China; ^3^Shenzhen College of Advanced Technology, University of Chinese Academy of Sciences, Shenzhen 518055, China; ^4^Dalian Medical College and University, Dalian 116044, China; ^5^Department of Zoology, Kohat University of Science and Technology, Kohat 26000, Pakistan; ^6^Department of Electrical Engineering, University of Science and Technology, Bannu 28100, Pakistan; ^7^Department of Information Technology, Faculty of Computing and Information Technology, King Abdulaziz University Jeddah, Saudi Arabia; ^8^College of Internet of Things (IoT) Engineering, Hohai University (HHU), Changzhou Campus, Nanjing 213022, China; ^9^Communication Research Laboratory, Department of Information and Communication Technology, Islamic University, Kushtia 7003, Bangladesh

## Abstract

Cancer has been found as a heterogeneous disease with various subtypes and aims to destroy the body's normal cells abruptly. As a result, it is essential to detect and prognosis the distinct type of cancer since they may help cancer survivors with treatment in the early stage. It must also divide cancer patients into high- and low-risk groups. While realizing efficient detection of cancer is frequently a time-taking and exhausting task with the high possibility of pathologist errors and previous studies employed data mining and machine learning (ML) techniques to identify cancer, these strategies rely on handcrafted feature extraction techniques that result in incorrect classification. On the contrary, deep learning (DL) is robust in feature extraction and has recently been widely used for classification and detection purposes. This research implemented a novel hybrid AlexNet-gated recurrent unit (AlexNet-GRU) model for the lymph node (LN) breast cancer detection and classification. We have used a well-known Kaggle (PCam) data set to classify LN cancer samples. This study is tested and compared among three models: convolutional neural network GRU (CNN-GRU), CNN long short-term memory (CNN-LSTM), and the proposed AlexNet-GRU. The experimental results indicated that the performance metrics accuracy, precision, sensitivity, and specificity (99.50%, 98.10%, 98.90%, and 97.50) of the proposed model can reduce the pathologist errors that occur during the diagnosis process of incorrect classification and significantly better performance than CNN-GRU and CNN-LSTM models. The proposed model is compared with other recent ML/DL algorithms to analyze the model's efficiency, which reveals that the proposed AlexNet-GRU model is computationally efficient. Also, the proposed model presents its superiority over state-of-the-art methods for LN breast cancer detection and classification.

The article "A Novel Hybrid Deep Learning Model for Metastatic Cancer Detection" was published in 2022. Journal: Comput Intell Neurosci.

## 1. Introduction

Cancer is a group of uncontrolled development cells in the body, which may spread to any organ abruptly [1, 2]. There are many distinct kinds of cancer, but lung cancer, breast cancer (BC), and skin cancer are the most prevalent. According to the World Health Organization (WHO) reports, the cancer death ratio is up to 9.2 million in lung cancer and 1.7 million in skin cancer, while breast cancer has caused 627,000 deaths [3, 4]. Breast cancer survival is strongly tied to the size of the tumor at the time of diagnosis; patients who have a tumor that is even less than 10 mm in size have a 98% chance of survival. When the tumor is 30 mm in size, 70% of breast cancer cases are diagnosed [5]. Therefore, the size of a breast tumor has a big impact on the detection and survival of a patient. There are so many imaging techniques used for the detection and classification of BC, such as X-ray [6], ultrasound [7], and CT scan [8]. Scientists use several methods to determine different kinds of cancer and present with symptoms, such as early-phase screening (EPS). In addition, they have developed unique approaches for the early identification of the prognosis in cancer treatment. Because of the invention of new technologies in medicine, vast volumes of cancer data have been collected and available for bioinformatics and the scientific community for evaluation and testing. However, the prediction of breast cancer disease is among the most fascinating and demanding challenges in healthcare, including incorrect classification by using these investigated diagnosis techniques.

Furthermore, a breast cancer diagnosis in clinics relies on pathologists' visual investigation of patients, who are highly qualified cancer specialists. However, this process is manual, which is a time-consuming and exhausting task that is very susceptible to human mistakes because most cells are usually a portion of irregular, arbitrary, and uncontrolled visual angles. It is important to determine whether a tumor is malignant or benign. The objective is to distinguish between the two classes. Since malignant tumors need early treatment because it is cancerous cell and spread abruptly. To limit and avoid future issues from occurring, the problem is a binary classification task to recognize malignant and benign issues that can be addressed using various machine learning and deep learning (ML/DL) algorithms [9–18]. The use of machine learning approaches to decrease the risk of developing cancer, recurrence, and survival prediction might increase the accuracy by 20% to 25% than last year [18]. However, handling high-dimensional and unbalanced data sets are challenging for ML methods.

The article "A Novel Hybrid Deep Learning Model for Metastatic Cancer Detection" was published in 2022. Journal: Comput Intell Neurosci.

To handle the above informative challenges, we have introduced a hybrid deep learning AlexNet gated recurrent unit (AlexNet-GRU) model to outperform a pathologist in terms of accuracy, precision sensitivity, and specificity of lymph node (LN) breast cancer detection. The following are the major contributions of this research:

- We have proposed a novel hybrid deep learning AlexNet-GRU model that automatically extracts features from the PCam data set and accurately identifies metastatic cancer
- The AlexNet-GRU classifier is used for successful metastatic cancer detection in clinical and biomedical research
- We have compared the performance of the proposed AlexNet-GRU model, the detection accuracy, and other performance metrics (precision, sensitivity, specificity, and time complexity) with the convolutional neural network GRU (CNN-GRU), CNN long short-term memory (CNN-LSTM) models, and other current ML/DL algorithms including state-of-the-art classification methods on the same data set to check the efficiency of the proposed model

The paper is organized as follows.  Section 2 provides the literature survey related to metastatic cancer detection. A framework for lymph node breast cancer detection, including explaining the experimental data set and data preprocessing, is presented in Section 3. A full discussion of the proposed model is given in Section 4. The experimental study of the hybrid model, including ML/DL methods with performance evaluation and discussion, is given in Section 5. Finally, the conclusion and future scope of the research are shown in Section 6.

## 2. Related Work

Various research has been done in metastatic cancer image classification, primarily to improve the evaluation performance of LN cancer detection. Previously, the classification of metastatic cancer images was investigated using several ML/DL approaches, including K-nearest neighbors (K-NN), support vector machines (SVM), convolutional neural networks (CNN), and so on. Sun et al. [19] used a graph-based method to classify breast cancer accurately and got an accuracy of 88.90% but had high time complexity (sec.), and they also compared SVM and K-NN algorithms. The comparative study indicated that SVM has high accuracy than K-NN in classifying LN breast cancer detection. Machhale et al. [20] introduced the CNNs model and achieved 89% accuracy in classifying malignant or benign cancer. Arunava [21] investigated the accuracy and error rate of K-NN and Naïve Bayesian methods of breast cancer classification and found that K-NN had better accuracy (85.90%) and lower error rate than Nave Bayesian approaches. Nawaz et al. [22] investigated CNN's approach to breast cancer detection. The method considered various types of breast cancer, and the results showed 88.4% accuracy.

The article "A Novel Hybrid Deep Learning Model for Metastatic Cancer Detection" was published in 2022. Journal: Comput Intell Neurosci.

In the research [23], Montazeri et al. created a rule-based method; they presented the classification of breast cancer and got accuracy up to 89% in the experimental study. Hossain and Rahaman [24] proposed a fuzzy logic method for categorizing bone cancers with 90.75% accuracy. A computer-aided approach [24] is also used to classify lung cancer that achieved an accuracy rate of 75.1%. Skin cancer classification was carried out using the visual geometry group NET (VGGNET) model, which was shown to be accurate at 78.66% [25]. The authors proposed a rough set technique for feature extraction and an SVM classifier for the breast cancer classification in women. They used a rough reduction technique to eliminate identical characteristics from the model to enhance accuracy. The authors in [25] proposed a rough set approach to extract features and an SVM classifier to classify breast cancer. They evaluated their proposed model's accuracy, sensitivity, and specificity by categorizing cancer images and comparing the results. Their findings showed that their method had the highest accuracy value of 92% and was more efficient than recent ML/DL models on the same data set. Aylin [26] presented a feature extraction method with a rough set method for breast cancer classification and an SVM classifier. They also implemented a rough reduction method to reduce unnecessary features from the model to improve accuracy and precision. In addition, the techniques mentioned above offer greater accuracy as compared to other investigated models. In addition, SVMs, artificial neural networks (ANNs), the K-NN, and various additional algorithms were used in breast cancer classification [26].

Saber et al. [27] proposed a deep learning model for automatic BC detection using the transfer learning method and six performance elevation matrices. For feature extraction and classification, they utilized five pretrained DL models, that is, Inception-V3, ResNet50, VGG19, VGG16, and Inception-V2 ResNet. The VGG16 model was shown to be effective for BC detection, with an accuracy of 98.96%. Togaçar et al. [28] presented a novel deep learning model for BC classification based on the concept of CNN. The model comprises two main parts. The hyper-column method attention component and the residual block are the two aspects of the model. When analyzing the BreakHis data set, the model achieves 98.80% accuracy. Ting et al. [29] proposed a new framework for BC classification named CNN improvement for BC classification (CNNI-BCC), using a supervised deep learning neural network to classify breast cancer. Experimental results showed that CNNI-BCC outperformed existing studies and attained an accuracy of 89.47%.

The article "A Novel Hybrid Deep Learning Model for Metastatic Cancer Detection" was published in 2022. Journal: Comput Intell Neurosci.

Eroglu et al. [30] proposed a CNN-based hybrid model for BC classification. The extracted features from breast cancer ultrasound images using AlexNet, ResNet50, MobileNetv2, and ResNet50. The extracted features are concatenated with the help of the mRMR method to increase accuracy. Finally, these features are classified with the SVM. The proposed hybrid model achieved 95.6% classification accuracy. Masud et al. [31] presented their own custom CNN model for BC detection. Moreover, they used eight pretrain, deep learning models for two BC data sets classification using a transfer learning strategy. The ResNet50 with Adam optimizer obtained the best accuracy of 92.4%, and VGG16 achieved the maximum AUC 0.97 score.

Another study [31] used AlexNet CNN's structure to detect mitosis images in breast histology and found 87% accuracy, and they compared performance metrics (sens, spec, and sens). The networks were capable of arranging the image in a pixel-by-pixel fashion. Gecer et al. [32] employed a DL technique to automatically identify and investigate the invasive ductal carcinoma (IDC) tissue zones and accurately detect cancer. Jason [33] demonstrated context-aware stacked CNNs for the classification of breast whole slide images (WSIs) into simple, DCIS (ductal carcinoma in situ), and IDC (in ductal carcinoma). The WSI classification achieved an area under the curve of 0.852 for classifying malignant and nonmalignant slides. In addition, the AlexNet CNN structure cannot store the memory of previous time-series patterns, where it is difficult to directly learn the most important and representative features of breast cancer that are given in the form of time series [34]. A GRU model is used with the AlexNet CNN structure to solve the above challenges. To improve the accuracy and other performance metrics (pres (%), sens (%), spec (%), and time complexity (sec) of classifications) [21, 35–42]. The literature related to this research is presented in Table 1.

## 3. A Framework for LN Breast Cancer Detection

This section proposes a new hybrid deep learning (AlexNet-GRU) model for metastatic (tumor) cancer detection and presents its framework, architecture, and classification performance evaluation. Besides, a conceptual representation of the entire classification scheme adopted in this study is shown in Figure 1 that consists of data collection, preprocessing, class labeling, model building, and evaluation for LN breast cancer detection.

The article "A Novel Hybrid Deep Learning Model for Metastatic Cancer Detection" was published in 2022. Journal: Comput Intell Neurosci.

### 3.1. Data Collection and Analysis

The cancer data set is obtained from the Kaggle [43]. The data set is an updated version of the original PCam data set, and there is no duplication within the data set. The collection contains 220,901 lymph node cancer images, with patches taken from 400 slide scan images from 162 women were LN breast cancer diagnosed and tested at University Medical Center, Netherlands. The first experimental training data set includes 170 WSIs samples of lymph node, and the second training data set consists of 100 WSIs. The data set contains high-resolution images (2,040 × 1,536 pixels). All the slides were scanned at 0.25 micro/pr using the same scanner to ensure consistency. Reduced-resolution images were sampled to a smaller region of pixel 50 × 50. It is organized into two main categories: metastatic tumors (cancer) and nonmetastatic (no-cancer) tumors, including 89,118 samples of LN breast cancer and 130,893 images of nonmetastatic tumors. The Kaggle data set is split into training data set 80% and testing 20% to avoid overfitting. Empirical studies show that the best results are obtained if we use 20–30% of the data for testing and the remaining 70–80% of the data for testing. The images are in the RGB color space and the PNG format.

Figure 2 presents the ratio of the cancerous photos and noncancer images. The training distribution of noncancerous/cancer was approximately 60/40.

### 3.2. Data Preprocessing

Preprocessing is very important for accurate classification performance. It is usually done on data before categorization. On the “cancer data set,” preprocessing methods are essential to enhance the model's classification accuracy. The most frequently utilized preprocessing methods are class labeling, picture scaling, data augmentation, random cropping, and sliding with the crop in breast cancer detection [44].

#### 3.2.1. Class Labeling

The cancer data set is subjected to the preprocessing method of class labeling that is conducted on the data set. The data set presentation of the class labeling is as follows: the label 0 for the image represents the patients who have no cancer (nonmetastatic cancer), while 1 represents the patient's “cancer” (metastatic cancer), as shown in Figure 3.

#### 3.2.2. Resizing

Resizing is another preprocessing method used in this study, as shown in Figure 4. The proposed model needs the same image size to obtain the desired results in the training process, so all the images were resized into identical dimensions.

The article "A Novel Hybrid Deep Learning Model for Metastatic Cancer Detection" was published in 2022. Journal: Comput Intell Neurosci.

#### 3.2.3. Data Augmentation

A data augmentation process was used in the cancer data set. Typically, a convolution neural network's structure performs better when working with big data, yet collecting vast amounts of data is challenging. Because of the limited quantity of data available, the convolution neural network suffers from an overfitting issue that reduces the performance evaluation of the models. The data augmentation approach is the most effective method of overcoming the underlying problem. The data augmentation of Kaggle cancer data sets is graphically shown in Figure 5.

#### 3.2.4. Random Cropping

An additional preprocessing method, namely random cropping with convolution neural networks (CNNs), was used to process the cancer data set. In the process of randomly cropping various sections large dimensional of images, the quantity of data available for the model needs significant data for training purposes.  Figure 6 presents the random cropping employed in the current study.

#### 3.2.5. Sliding with Crop

In sliding with the crop process, initially, the images of the PCam data set were cropped. To increase the number of images, they should be arranged from left to right and top to bottom to handle the overfitting issue.  Figure 7 shows sliding with the crop process.

#### 3.2.6. Row Major Order

Multi-dimensional arrays of images are stored in one dimension or a single row when they are stored in row-major order. Images may be in greyscale or RGB format, depending on their size. Greyscale images are composed of two channels, including white and black. RGB pictures are three channels: green, red, and blue. RGB images are more complex than greyscale pictures. The row-major order is shown in Figure 8.

## 4. Proposed System Model

After preprocessing steps, the next section is to feed data into the proposed model (AlexNet-GRU). This section introduces the AlexNet and GRU model, including training parameters for lymph node (LN) breast cancer detection and classification.

### 4.1. AlexNet Model

The AlexNet is the submodel of CN that has made significant contributions, particularly in applying objection detection, image classification, and so on. It had won the Image Net LSVRC-2012 competition by a considerable margin (15.3% error rates vs. 26.2% error rates in second place). The network's design was very similar to that of the LeNet network. However, it was deeper, had more filters per layer, and featured convolutional layers. It was composed of convolutions, max pooling, ReLU activations, and dropout layers.  Figure 9 describes the basic structure of the AlexNet model. The following steps present the mathematical formula of the AlexNet model as follows.

The article "A Novel Hybrid Deep Learning Model for Metastatic Cancer Detection" was published in 2022. Journal: Comput Intell Neurosci.

#### 4.1.1. Convolution Layers

The convolution layer is the main building block of the AlexNet model. It consists of different learnable filters that extract the input data features. The feature map assumes that the *c*^th^ of layer *d* is represented by *y*_*c*_^*d*^ and that the *J*^th^ at layer *d* – 1 is represented by *y*_*c*_^*d*−1^. The value of *y*_*c*_^*d*^ is calculated as follows:

(1) $$\begin{array}{c} y_{c}^{d}=\sum_{j\in bc}k_{cj}^{d}*y_{\dot{J}}^{d-1}+a_{c}^{d}, \end{array}$$

where |b| is the number of mapping features at layer *d*, *a*_*c*_^*d*^ is a biased term distributed throughout all connections to the *c* feature map, and *b*_*c*_ is a subset of feature maps in layer *d* − 1 related to units *c*, at layer *d*.

#### 4.1.2. Activation Function (ReLU_Func)

The activation *d*(*y*) of ReLU_Func can be expressed as follows:

(2) $$\begin{array}{c} d\left(y\right)=\max\left(0,y\right), \end{array}$$

where the range value is from 0 to *y*.

#### 4.1.3. Max_Pooling

The max_pooling can be mathematically represented as follows:

(3) $$\begin{array}{c} y_{c^{\left(d+1\right)}}j^{d+1},r=\underset{0\leq c<G,0\leq j<C}{\max}x_{c^{d+1}}^{d}*G+i,j^{d+1}*W+j, \end{array}$$

where

(4) $$\begin{array}{c} 0\leq f^{d+1}<g^{d+1},0\leq j^{d+1}<W^{d+1},0\leq d<D^{d+1}=D^{d}. \end{array}$$

A triplet (*c*^*d*^, *J*^*d*^, *d*^*d*^) finding one component in the input *x*^*d*^ and another triplet (*c*^*d*+1^, *J*^1+1^, *d*^*d*+1^) to determine the location of one component inside *y* are needed. The pooling output *y*_*c*^(*d*+1)^_*j*^*d*+1^, *d* comes from *x*_*c*^*l*,*j*^*d*^,*d*^*d*^^_^*d*^ with the given condition is true. The (*c*^*d*^, *j*^*d*^) − *th* distinct entry belongs to the (*c*^*d*+1^, *j*^*d*+1^)^th^ subregion.

#### 4.1.4. Forward Pass of CNN

The forward pass of a CNN may be expressed mathematically as follows:

(5) $$\begin{array}{c} c^{1}⟶d^{1}⟶c^{2}⟶\ldots C^{K-1}⟶d^{k-1}⟶C^{K}⟶d^{K}⟶E. \end{array}$$

The forward pass of the CNN layer is shown in equation (5). Here, *c*^1^, *c*^*K*−1^, and *c*^*K*^ are the CNNs, *c*^1^, *d*^*K*−1^, *d*^*K*^ show the layer processing, and *E* expresses the cost function. Let us assume that *j* presents the actual value, while *c*^*K*^ represents the cost function values can be mathematically expressed as follows:

(6) $$\begin{array}{c} E=\frac{1}{2}{\left\|j-c^{k}\right\|}^{2}. \end{array}$$

### 4.2. Gated Recurrent Unit Network

The GRU model was most often employed in recurrent neural networks (RNN) to address the vanishing gradient issue, as shown in Figure 10. In comparison to LSTM, GRU has three major gates and an internal cell state, making it more efficient. The information is stored in a secret state inside the GRU. The backward and forward information is provided with the update gate (*z*), whereas the previous knowledge is presented in the reset gate (*r*). The current memory gate uses the reset gate to preserve and keep the required information from the previous state of the computer. With the input modulation gate, it is possible to introduce nonlinearity into the input while also providing it with the characteristics of a zero-mean. According to the following definition, the mathematical description of the fundamental GRU of rest and updated gates is

(7) $$\begin{array}{c} r_{t}=\sigma \left(X_{t}.W_{xr}+H_{t-1}.W_{hr}+b_{r}\right),\\ Z_{t}=\sigma \left(X_{t}.W_{xz}+H_{t-1}.W_{hz}+b_{z}\right), \end{array}$$

where *W*_*rx*_ and *W*_*xz*_ are weight parameters and *b*_*r*_ and *b*_*z*_ represent biased.

The article "A Novel Hybrid Deep Learning Model for Metastatic Cancer Detection" was published in 2022. Journal: Comput Intell Neurosci.

### 4.3. AlexNet-GRU Model

In this research, we propose the AlexNet-GRU model for breast cancer classification. The proposed model is composed of seven convolutions, four max-pooling, three completely linked layers, and ReLU as an activation function. The proposed AlexNet-GRU model's structure and employed parameters are shown in Figure 11 and Table 2, respectively.

Initially, the input shape of the image was (60, 60, 3) size, where the image height was 60 pixels and width 60 pixels with RGB, and the number of channels was 3.

To extract the features from the input shape, it passes through the first convolutional layer of the proposed model, where the output shape of the feature map was 128. Additionally, the stride and the kernel size of the convolutional layer were (3 × 3) and 1. While padding was the same for all of the layers of the proposed model and rectified linear units (ReLU) were used as activation function to decrease the nonlinearity dimension problem, followed by conventional layer 1. After the convolutional layer 1, the output shape contained (60, 60) size and 128 feature maps. The pooling layer decreases the training parameter up to (58, 58) size that speeds up the process of the proposed model. After the pooling layer, the training parameter (58, 58, 128) were passed through drop_out to prevent the model from overfitting issues. An initial dropout of 0.9 was used in the convolution layer to avoid the overfitting problem. After each conventional and max-pooling layer, the training parameter was substantially decreased, followed by activation function (ReLU) and drop out. After the training process of the traditional and max-pooling layers, the data must be composed into an ID array to use as input for a fully connected layer implemented by flatten with training parameters (42, 42) size and features map (512) had been produced. After completing all the convolutional layers process, the dropout was used that made 1,024 feature maps. A GRU model was employed with a fully connected layer composed of 1,024 neurons to solve the vanishing gradient problem. After the GRU model, two fully connected layers were also used. Finally, SoftMax operations were implemented with the final linked layer.

The article "A Novel Hybrid Deep Learning Model for Metastatic Cancer Detection" was published in 2022. Journal: Comput Intell Neurosci.

## 5. Performance Evaluation and Discussion

This section presents the classification performance (accuracy, precision, sensitivity, and specificity), including experimental setup and enhanced comparative study of the proposed model (AlexNet-GRU) with CNN-GRU, CNN-LSTM, and the recent ML/DL models for lymph node breast cancer detection.

### 5.1. Experimental Setup

We have utilized an Intel Core i6 processor and a graphics-processing unit (GPU) from NVIDIA for this experiment. The proposed model has also been trained by merging Keras with the Python 3.8 programming environment. Detailed descriptions of the employed software and hardware characteristics are presented in Table 3.

### 5.2. Performance Metrics

The performance metrics are taken into consideration to evaluate the proposed model's viability and to distinguish between breast cancer (tumor) and normal tissue properly, such as the following:

TP: The cancer samples were positive

TN: It refers to negative (noncancer) samples

FP: It presents negative but is predictable to be positive

FN: It presents positive samples predictable to be negative by the model

The mathematical representations of the accuracy, precision, sensitivity, and specificity that are used as performance metrics to identify cancer in most cases are as follows:

(8) $$\begin{array}{c} Acc\left(\%\right)=\frac{\text{TruePostive}\left(\text{TF}\right)+\text{TrueNegative}\left(\text{TN}\right)}{\text{TruePostive}\left(\text{TP}\right)+\text{TrueNagative}\left(\text{TN}\right)+\text{FalsePostive}\left(\text{FP}\right)+\text{FalseNegative}\left(\text{FN}\right)},\\ \mathrm{Pr}ec\left(\%\right)=\frac{\text{TruePostive}\left(\text{TP}\right)}{\text{TruePostive}\left(\text{TP}\right)+\text{FalsePostive}\left(\text{FP}\right)},\\ Sen\left(\%\right)=\frac{\text{TruePostive}\left(\text{TP}\right)}{\text{TruePostive}\left(\text{TP}\right)+\text{FalseNegative}\left(\text{FN}\right)},\\ Spec\left(\%\right)=\frac{\text{TrueNegative}\left(TN\right)}{\text{TrueNegative}\left(\text{TN}\right)+\text{FalsePostive}\left(\text{FP}\right)}. \end{array}$$

The article "A Novel Hybrid Deep Learning Model for Metastatic Cancer Detection" was published in 2022. Journal: Comput Intell Neurosci.

### 5.3. Accuracy, Precision, Sensitivity, and Specificity

This study introduced three models, CNN-GRU, CNN-LSTM, and the proposed AlexNet-GRU model, to compare cancer image classification. Every model has two classes, such as 0 and 1. The result indicates that the proposed model exhibits the best accuracy, precision, sensitivity, and specificity, while CNN-GRU shows the lowest performance in terms of performance metrics, as shown in Figure 12.  Table 4 shows the experimental results of the employed models' accuracy, precision, sensitivity, and specificity.

### 5.4. Receiver-Operating Characteristic (ROC) Analysis

The ROC is an experimental tool to express the diagnostic tests' evaluation performance or the ratio of sensitivity and 1-specificity. The ROC of the proposed AlexNet-GRU model, CNN-LSTM, and CNN-GRU of the binary class recognition task of breast cancer detection is shown in Figure 13. The ROC indicates that the proposed model accurately classifies metastatic cancer (tumor or cancer) and nonmetastatic cancer (no cancer) of lymph nodes compared to CNN-LSTM and CNN-GRU models.

### 5.5. Time Complexity (ms)

This section represents the time complexity of the models based on the testing. Because the training is performed mostly offline and not considered in the evaluation process. Furthermore, the testing technique is viewed as a critical statistic since it reveals the efficiency and general performance, important performance indicators. On the breast cancer detection task, the proposed AlexNet-GRU model is time-efficient for binary class recognition tasks compared to CNN-GRU and CNN-LSTM models, as shown in Figure 14.

Performance metrics are compared with existing deep learning algorithms, such as CNN, deep neural network (DNN), LSTM, GRU, and BiLSTM for binary tasks to demonstrate the efficiency of the proposed AlexNet-GRU model for binary tasks. As shown in Figure 15, the findings reveal that all of the current deep learning algorithms are less accurate (%) than the proposed model, while CNN and LSTM are the least accurate models among all of the models. In Table 5, the proposed model's performance is compared to the state-of-the-art ML/DL algorithms for the BC classification task.

The proposed model shows better performance accuracy (%). However, the proposed model has some disadvantages. The AlexNet-GRU method has high time complexity (ms) and requires high computational power and specialized hardware such as a good GPU to expedite the training process.

Recently, there also exist some other artificial intelligence technologies that can be used in next-generation healthcare systems, that is, federated learning algorithms [52], deep learning algorithms [53], reinforcement, and deep reinforcement learning algorithms [54–58]. In addition, next-generation industries, that is, Industry 4.0 and Industry 5.0, would play a crucial role in developing advanced equipment used in health treatment [59].

The article "A Novel Hybrid Deep Learning Model for Metastatic Cancer Detection" was published in 2022. Journal: Comput Intell Neurosci.

## 6. Conclusions

This research intended to classify lymph node breast cancer detection using the proposed Alex net-GRU model. To train the model, the preprocessing step was done by using various types of techniques to achieve the best classification performance. Furthermore, the experimental study was performed with CNN-GRU, CNN-LSTM, and recent ML/DL models. We used a well-known Kaggle (PCam) data set to classify lymph node cancer samples. The experimental results indicated that the performance metrics accuracy, precision, sensitivity, and specificity (99.50%, 98.10%, 98.90%, and 97.50%) of the proposed model can reduce the pathologist errors made during the diagnosis process of incorrect classification and significantly better performance than CNN-GRU and CNN-LSTM models. To analyze the model efficiency, the proposed model was compared with recent ML/DL algorithms that revealed that the proposed AlexNet-GRU model is computationally efficient and outperformed. Also, the proposed model presented its superiority over state-of-the-art methods for breast cancer detection and classification. The proposed AlexNet-GRU model showed about 3% best accuracy and other performance metrics. Therefore, the presented AlexNet-GRU model is a promising technique for categorizing lymph node breast cancer detection and classification. This research can be further expanded by adding one or more layers with the AlexNet-GRU model and will be tested on multi-classification breast cancer detection and not limited to binary recognition tasks.

## Figures and Tables

**Figure 1:** The basic block diagram of the AlexNet-GRU model for lymph node (LN) breast cancer detection.

**Figure 2:** The ratio of malignant (cancerous images) and benign (noncancer images).

**Figure 3:** Breast images of metastatic cancer and non-metastatic.

**Figure 4:** Resizing technique for breast cancer image data set.

**Figure 5:** Data augmentation for breast cancer data set.

**Figure 6:** Random cropping of the breast cancer data set.

**Figure 7:** Sliding with a crop of the breast cancer image data set.

**Figure 8:** Row major order of the breast cancer image data set.

**Figure 9:** Structure of the AlexNet model.

**Figure 10:** The basic structure of the GRU model.

**Figure 11:** The general structure of the proposed AlexNet-GRU model.

**Figure 12:** The classification performance of the proposed AlexNet-GRU, CNN-GRU, and CNN-LSTM models for binary recognition task of BC detection.

The article "A Novel Hybrid Deep Learning Model for Metastatic Cancer Detection" was published in 2022. Journal: Comput Intell Neurosci.

**Figure 13:** The ROC performance of the given models: (a) proposed AlexNet-GRU, (b) CNN-GRU, and (c) LSTM-GRU.

**Figure 14:** The time complexity (ms) of the binary BC detection.

**Figure 15:** The classification performance comparison of the proposed model with other existing DL models in BC detection.

**Table 1:** The literature employed ML/DL models for breast cancer detection.

Publication	Algorithms	Data set	Detection accuracy (%)	Time complexity (ms)
[35]	RF, K-NN	UCI-cancer	87%, 88%	N/A
[36]	DNN	BCW (breast cancer Wisconsin)	75%	High
[37]	DCNN, CNN	BreakHis	90%, 90.1%	High
[21]	CNN	MIAS	90%	High
[38]	RF, SVM, K-NN	UCI-cancer WBCD11, WBCD32	76%, 75%, 74%	N/A
[39]	DNN	BCW (breast cancer Wisconsin)	79.01%	High
[40]	SVM, RF, K-NN	BCW (breast cancer Wisconsin)	77%, 74%, 75%	High
[41]	GRU, RNN	UCI-cancer	78.90%	N/A
[42]	CNN	BCW (breast cancer Wisconsin)	70.50%	High

**Table 2:** Training parameters of the proposed AlexNet-GRU model.

Layers	K_Size	Input (shape)	Act_Func	Output (shape)
Con_Layer_1	3 × 3	(60, 60, 3)	ReLU_Func	(58, 58, 128)
B-Norm_1	—	(58, 58, 128)	—	(58, 58, 128)
Max_pooling_1	2 × 2	(58, 58, 128)	—	(57, 57, 128)
Drop_out = 0.9	—	(57, 57, 128)	—	(57, 57, 128)
Con_Layer_2	2 × 3	(57, 57, 128)	ReLU_Func	(55, 55, 256)
B-Norm_2	—	(57, 57, 128)	—	(55, 55, 256)
Max_pooling_2	2 × 2	(55, 55, 256)	—	(54, 54, 256)
Drop_out = 0.9	—	(54, 54, 256)	—	(54, 54, 256)
Con_Layer_3	2 × 3	(54, 54, 256)	ReLU_Func	(52, 52, 256)
B-Norm_3	—	(52, 52, 256)	—	(52, 52, 256)
Max_pooling_3	2 × 2	(52, 52, 256)	—	(51, 51, 256)
Dropout = 0.5	—	(51, 51, 256)	—	(51, 51, 256)
Con_Layer_4	2 × 3	(51, 51, 256)	ReLU_Func	(49, 49, 256)
B-Norm_4	—	(49, 49, 256)	—	(49, 49, 256)
Dropout = 0.9	—	(49, 49, 256)	—	(49, 49, 256)
Con_Layer_5	2 × 3	(49, 49, 256)	ReLU_Func	(47, 47, 256)
B-Norm_5	—	(47, 47,256)	—	(47, 47, 256)
Dropout = 0.9	—	(47, 47, 256)	—	(47, 47, 256)
Con_Layer_6	2 × 3	(47, 47, 256)	ReLU_Func	(45, 45, 256)
B-Norm_6	—	(45, 45, 256)	—	(45, 45, 256)
Dropout = 0.9	—	(45, 45, 256)	—	(45, 45, 256)
Con_Layer_7	2 × 3	(45, 45, 256)	ReLU_Func	(45, 45, 512)
B-Norm_7	—	(43, 43, 512)	—	(43, 43, 512)
Max_pooling_4	3 × 2	(43, 43, 512)	—	(42, 42, 512)
Dropout = 0.5	—	(42, 42, 512)	—	(42, 42, 512)
Flatten	—	(42, 42, 512)	—	(903,168)
Dense1	—	(903,168)	—	(1,024)
B-Norm_8	—	(1,024)	—	(1,024)
Drop_out = 0.3	—	(1,024)	—	(1,024)
Dense2	—	(1,024)	—	(2,000)
B-Norm_9	—	(2,000)	—	(2,000)
GRU		(1,024)	—	—
Dense3	—	(2,000)	—	(2,000)

**Table 3:** The experimental setup.

GPU	1,060 6 GB, Nvidia GeForce
CPU	Core-i6, 6th Generation, and 2.80 GHz processor
RAM	16 GB
Operating system	Windows 64 bit
Libraries	Pandas, NumPy, Scikit-learn, TensorFlow, and Keras
Languages	Python 3.7

The article "A Novel Hybrid Deep Learning Model for Metastatic Cancer Detection" was published in 2022. Journal: Comput Intell Neurosci.

**Table 4:** The experimental results of the proposed AlexNet-GRU, CNN-GRU, and CNN-LSTM models for BC image classification.

Performancemetrics (%)	Classification	CNN-GRU (%)	CNN-LSTM (%)	Proposedmodel (%)	Data set	Other parameters
Accuracy (%)	Binary class	97.10	97.90	**99.10**	Kaggle	Batch size = 100,epoch = 100, optimizer = Adam
Precision (%)		96.90	97.70	**98.70**		
Sensitivity (%)		96.87	97.60	**98.71**		
Specificity (%)		96.59	97.10	**98.51**		

**Table 5:** Comparative study of the proposed model with recent ML/DL models.

Publication	Cancer type	Models	Classification type	Data set	Accuracy (%)
[45]	Breast cancer	ANN	Binary class	SNPs	69%
[46]	Colon carcinomatosis	BN	Binary class	Clinical, pathologic	71%
[47]	Multiple myeloma	SVM, DCNN	Multi-class	DDSM (CBIS-DDSM)	71%, 93%
[48]	Breast cancer	DCNNs	Bi-multi-class	Kaggle	90%, 93%
[49]	Breast cancer	DCNNs	Multi-class	Wisconsin diagnostic breast cancer (WDBC)	88%
[50]	Breast cancer	ResNet	Multi-class	Kaggle	85%
[51]	Breast cancer	Pretrained CNN	Binary class	Kaggle	90%
Proposed model	Breast cancer	AlexNet-GRU	Binary class	Kaggle	99.50%

## Data Availability

The data are publicly available at https://www.kaggle.com/c/histopathologic-cancer-detection/data.
